# Prediction Model of Postoperative Severe Hypocalcemia in Patients with Secondary Hyperparathyroidism Based on Logistic Regression and XGBoost Algorithm

**DOI:** 10.1155/2022/8752826

**Published:** 2022-07-25

**Authors:** Chao Ding, Yuwen Guo, Qinqin Mo, Jin Ma

**Affiliations:** ^1^Hemodialysis Room, Department of Renal Endocrinology, Anhui Lujiang People's Hospital, Lujiang 231501, China; ^2^Department of Renal Endocrinology, Anhui Lujiang People's Hospital, Lujiang 231501, China; ^3^Department of Geriatric Medicine, The First People's Hospital in Hefei, Hefei 230061, China

## Abstract

**Objective:**

A predictive model was established based on logistic regression and XGBoost algorithm to investigate the factors related to postoperative hypocalcemia in patients with secondary hyperparathyroidism (SHPT).

**Methods:**

A total of 60 SHPT patients who underwent parathyroidectomy (PTX) in our hospital were retrospectively enrolled. All patients were randomly divided into a training set (*n* = 42) and a test set (*n* = 18). The clinical data of the patients were analyzed, including gender, age, dialysis time, body mass, and several preoperative biochemical indicators. The multivariate logistic regression and XGBoost algorithm models were used to analyze the independent risk factors for severe postoperative hypocalcemia (SH). The forecasting efficiency of the two prediction models is analyzed.

**Results:**

Multivariate logistic regression analysis showed that body mass (OR = 1.203, *P* = 0.032), age (OR = 1.214, *P* = 0.035), preoperative PTH (OR = 1.026, *P* = 0.043), preoperative Ca (OR = 1.062, *P* = 0.025), and preoperative ALP (OR = 1.031, *P* = 0.027) were positively correlated with postoperative SH. The top three important features of XGBoost algorithm prediction model were preoperative Ca, preoperative PTH, and preoperative ALP. The area under the curve of the logistic regression and XGBoost algorithm model in the test set was 0.734 (95% CI: 0.595~0.872) and 0.827 (95% *CI*: 0.722~0.932), respectively.

**Conclusion:**

The predictive models based on the logistic regression and XGBoost algorithm model can predict the occurrence of postoperative SH.

## 1. Introduction

Secondary hyperparathyroidism (SHPT) is a common complication in patients with chronic renal insufficiency [1]. It refers to the syndrome caused by the excessive secretion of parathyroid hormone (PTH) stimulated by low blood calcium or high blood phosphorus for various reasons and is one of the common severe complications of maintenance hemodialysis patients [2, 3]. The main manifestations of SHPT patients are elevated parathyroid hormone, calcium and phosphorus metabolism disorder, ectopic calcification, and osteoporosis [4]. About 50% of the death causes of dialysis patients are cardiovascular events caused by vascular calcification, which seriously affects patients' quality of life and survival time [5].

Treatment of SHPT includes the normalization of serum phosphorus and calcium levels and optimization and improvement of parathyroid hormone levels [6, 7]. For patients with SHPT who are refractory to treatment or cannot afford expensive drugs, parathyroidectomy (PTX) can quickly and effectively control PTH levels and prevent progression [8, 9]. However, after PTX, serum calcium (Ca), phosphorus (P), and parathyroid hormone levels were significantly reduced [10]. A sudden drop in parathyroid hormone leads to a brief and significant increase in bone remineralization, with rapid transfer of calcium from the circulation to bone tissue [11]. Patients with mild clinical symptoms may be accompanied by weakness, headache, and paresthesia [12]. Severe postoperative hypocalcemia (SH) is the most common complication after PTX, with an incidence of 70%-97%, and patients can develop life-threatening complications [13].

SH in patients is a common complication after PTX. How to effectively prevent and correct SH is the main concern after PTX. At present, there are few studies on the risk factors related to SH after PTX. Building machine models to predict diseases has become a hot topic in recent years [14]. In this study, the XGBoost algorithm and logistic regression model were used to analyze the influencing factors of calcium demand after SHPT and to provide therapeutic strategies for postoperative correction of postoperative SH.

## 2. Material and Methods

### 2.1. General Data

A total of 60 patients diagnosed with SHPT who underwent SHPT in our department from January 2017 to December 2019 were retrospectively selected as the study subjects. The inclusion criteria of 60 patients have met the Improving Global Outcomes (KDIGO) for the Diagnosis, Evaluation, Prevention, and Treatment of Chronic Kidney Disease-Mineral and Bone Disorder (CKD-MBD): (1) PTH > 800 pg/mL and (2) chronic renal insufficiency [15]. All patients had the following surgical indications: severe SHPT symptoms, such as hyperphosphatemia, postoperative SH, pruritus, and bone pain. None of the 60 patients had severe cardiac insufficiency. Exclusion criteria include complicated with other serious diseases and complications and poor treatment compliance.

### 2.2. Study and Analyze Variables

General data and laboratory results of patients were included in the analysis. General data of the patients include gender, age, body mass, dialysis time, and parathyroid gland volume. Laboratory examination included intact serum parathyroid hormone (PTH), serum calcium (Ca), serum phosphorus (P), and serum alkaline phosphatase (ALP) from preoperative patients.

### 2.3. Construction of Logistic Regression Model

Logistic regression is a commonly used statistical learning model to predict the outcome of binary variables. The dependent variable *y* is a dichotomous variable and only takes 0 and 1. *P* = *P*(*y* = 1|*x*_1_, ⋯, *x*_*k*_) is the object of study, It is affected by *K* factors and is called binary logistic linear regression model or logistic regression model for short.

(1) $$\begin{array}{c} \ln\frac{P}{1-P}=\beta_{0}+\beta_{1}x_{1}+\cdots +\beta_{k}x_{k}. \end{array}$$

The value *P*/(1 − *P*) = *e*^*β*_0_+*β*_1_*x*_1_+⋯+*β*_*k*_*x*_*k*_^ of the advantage ratio *P*/(1 − *P*) can be obtained from formula (1). The calculation formula of *P* can be obtained:

(2) $$\begin{array}{c} P=\frac{e^{\beta_{0}+\beta_{1}x_{1}+\cdots +\beta_{k}x_{k}}}{1+e^{\beta_{0}+\beta_{1}x_{1}+\cdots +\beta_{k}x_{k}}}. \end{array}$$

### 2.4. Construction of XGBoost Algorithm Model

XGBoost reduces the complexity of the model and avoids overfitting by adding regularization terms into the objective function on the basis of gradient lifting decision tree. The objective function is

(3) $$\begin{array}{c} \text{Obj}=\underset{i}{\sum }l\left({\hat{y}}_{i},y_{i}\right)+\underset{k}{\sum }\text{Ո}\left(f_{k}\right)+C, \end{array}$$

(4) $$\begin{array}{c} \text{Ո}\left({\text{f}}_{\text{k}}\right)=\gamma T+\frac{1}{2}\lambda {\left\|\text{w}\right\|}^{2}=\gamma T+\frac{1}{2}\lambda \overset{\text{T}}{\underset{\text{j}=1}{\sum }}{\text{w}}_{\text{j}}^{2}. \end{array}$$

*γ* and *λ* are the penalty coefficient for the model. *T* and *w* represent the number of leaves and the weight of leaves in the *K*th tree, respectively. *c* is a constant term. XGBoost performs second-order Taylor expansion on this basis, assuming that the loss function of the *t* time is defined as

(5) $$\begin{array}{c} {\text{Obj}}^{\left(t\right)}=\underset{i}{\sum }l\left({\hat{y}}_{i}^{t-1},y_{i}+f_{t}\left(x_{i}\right)\right)+\text{Ո}\left(f_{t}\right). \end{array}$$

Second-order Taylor expansion is performed on formula (4), and the constant term is simplified and removed:

(6) $$\begin{array}{c} {\text{Obj}}^{\left(t\right)}=\overset{n}{\underset{i=1}{\sum }}\left[g_{i}f_{t}\left(x_{i}\right)+\frac{1}{2}h_{i}f_{t}{\left(x_{i}\right)}^{2}\right]+\text{Ո}\left(f_{t}\right). \end{array}$$

### 2.5. Establishment of Study Sequence

The data sets of SHPT patients were randomly divided into a training set (*n* = 42) and a test set (*n* = 18) based on a 7 : 3 ratio. The training set is used to fit the prediction model, and the test set is used to evaluate the model effect. To prevent overfitting and improve the model's prediction performance, the independent risk factors of postoperative SH were analyzed by one-way ANOVA and Mann–Whitney *U* test in the logistic regression prediction model, and the optimal model in the training set was screened. Regression coefficient, OR value, and 95% CI can reflect the effects of predictors in the logistic prediction model (Figure 1).

In the XGBoost prediction model, parameters are firstly adjusted by adjusting the weight of the leaf node and the depth of the tree model. Then, the training set was further subdivided into 10 pieces using the 10-fold cross-validation method. One of them was cyclically extracted as the verification set to adjust the hyperparameters of XGBoost. In the XGBoost prediction model, the importance of the predictors is reflected by the important feature score (Figure 2). The patients in the training set were divided into the SH group and nonsevere hypocalcemia (non-SH group) according to postoperative blood calcium level. According to the quality guidelines for prognosis of renal disease, blood calcium < 1.8 mmol/L 7 days after the operation was defined as the SH group. In contrast, serum calcium > 1.8 mmol/L 7 days after the operation was defined as the non-SH group [16].

### 2.6. Statistical Analysis

The Shapiro-Wilk test is performed to determine the normality of the data. The measurement data conforming to normal distribution were described by mean ± standard deviation. SPSS 20.0 software was used for statistical analysis. The predictive effectiveness of the logistic regression model and the XGBoost algorithm model was evaluated with the receiver characteristic curve (ROC). The larger the area under the curve is, the higher the prediction efficiency will be. *P* < 0.05 means the difference is statistically significant.

## 3. Results

### 3.1. Comparison of Clinical Data

Among the 42 patients in the training set, 25 were male and 17 were female. The mean age of the patients was 49.6 ± 7.8 years. Of the 18 patients in the test set, 11 were male and 7 were female. The patient's age was 48.7 ± 6.9 years. There were no significant differences in gender, age, body weight, dialysis time, and parathyroid gland volume between the training set and the test set (*P* > 0.05). The specific data are shown in Table 1.

### 3.2. Comparison of Clinical Data between the SH Group and Non-SH Group

Patients in the training group were divided into the SH group (*n* = 18) and the non-SH group (*n* = 24) according to postoperative blood calcium levels. There were no significant differences between the two groups in terms of gender, dialysis time, parathyroid gland volume, and preoperative serum P (*P* > 0.05). However, there were statistically significant differences in age, body weight, preoperative PTH, preoperative Ca, and preoperative ALP between the two groups (*P* < 0.05). Detailed information is shown in Table 2 and Figure 3.

### 3.3. Logistic Regression Analysis Results

Multivariate logistic regression analysis showed that body mass, preoperative PTH, and preoperative ALP were positively correlated with postoperative SH, which were risk factors. However, age and preoperative Ca were negatively correlated with postoperative SH, which were protective factors (Table 3).

### 3.4. Important Feature Score of XGBoost Model

The variables in the training set are incorporated into the algorithm model for training, and the scoring results of important features are finally obtained. According to the score, the order is preoperative Ca, preoperative PTH, preoperative ALP, age, and body mass. The important feature scores in the XGBoost algorithm model are shown in Figure 4.

### 3.5. Evaluation of the Effectiveness of Prediction Models

The area under the curve of the logistic regression model in the training set was 0.754 (95% CI: 0.619~0.888), and the area under the curve of the XGBoost algorithm was 0.784 (95% CI: 0.655~0.913). The area under the curve of the logistic regression model in the test set was 0.734 (95% CI: 0.595~0.872), and the area under the curve of the XGBoost algorithm was 0.827 (95% CI: 0.722~0.932). The ROC is shown in Figure 5.

## 4. Discussion

The SHPT is a common complication of maintenance dialysis patients, which can cause symptoms such as dialysis bone pain, pruritus, and insomnia and even significantly increase the fatality rate [17]. PTX is the most important treatment for patients with refractory SHPT [8]. Postoperative SH is a common postoperative complication of SHPT patients. Patients may experience convulsions of the limbs, numbness, laryngeal muscle spasm, and even cardiac arrest, which is a difficulty in the current treatment [4]. Therefore, it is of great clinical significance to explore the influencing factors of SHPT after PTX to prevent and treat SH.

The mechanism of SH occurrence after PTX is that PTH in postoperative blood circulation decreases rapidly and 2 hours after surgery is often reduced to less than 10% of the preoperative level. This causes a decrease in intestinal calcium absorption and slows down osteoclasts. The rapid deposition of serum Ca and serum P into the bone tissue leads to a sharp drop in blood Ca levels, presenting as persistent and SH, also known as “bone starvation” syndrome [18]. Several studies have shown that the incidence of severe SH after PTX is 70%~90% [19].

According to the study, age, body weight, preoperative PTH, preoperative Ca, and preoperative ALP have statistical significance with postoperative SH (*P* < 0.05). In this study, the logistic regression model was used to analyze and show that age, body weight, preoperative PTH, preoperative Ca, and preoperative ALP have an impact on postoperative SH. In addition, the XGBoost algorithm model is also constructed in this study, and the top three variables are preoperative Ca, preoperative PTH, and preoperative ALP according to important feature scores, while preoperative Ca level is a protective factor for postoperative SH. Many previous studies have confirmed the influence of preoperative Ca on postoperative SH [20, 21]. PTH is one of the main hormones regulating Ca and P metabolism in the body. After PTX, PTH level decreases rapidly, intestinal Ca absorption decreases, osteogenesis rate exceeds osteolysis, and blood Ca deposits to the bone tissue, so blood Ca decreases significantly [22]. ALP is a recognized biomarker of renal osteodystrophy [23]. The sudden decrease of PTH in SHPT patients after surgery can affect osteoclast activity and bone resorption, leading to postoperative SH and the corresponding increase in serum ALP level [24]. PTH regulates the balance of serum Ca and serum P, promotes bone resorption, and inhibits bone formation. Our study was similar to previous studies. Yang et al. [25] showed that preoperative ALP affected postoperative SH. The higher the preoperative ALP level of PTX was, the more obvious postoperative SH would be.

In addition, based on multiple logistic regression, our study also found that age and body mass were also related variables of postoperative SH, among which age was negatively correlated with postoperative low Ca. Based on the XGBoost algorithm prediction model, it was found that although body mass was the influencing factor of SH after PTX, it had the lowest feature score. Ge et al. recently found that patients with higher body mass have higher bone mass and hence greater postoperative total Ca requirements [26]. These results indicate that monitoring and managing body mass are of great significance in preventing and treating SH after an operation. Recent studies have shown that body mass is an independent predictor of SH, and overweight and obesity are risk factors for SH [27].

Logistic regression is one of the most commonly used statistical models in which the outcome variables are dichotomous [28]. The XGBoost algorithm model can not only control the complexity of the model but also prevent the model from overfitting due to the regular term added into the loss function [14]. In this study, the prediction models of postoperative SH in patients with SHPT based on logistic regression and XGBoost algorithm have good prediction efficiency.

This study has some limitations. First, not many predictive variables are included in this study, which may affect the prediction results. Second, the relatively small sample size may mask potentially significant associations between variables. Therefore, increasing the predictive variables and the sample size is the focus of future research. In the future, more algorithms will be tried to predict postoperative SH [29–31].

## 5. Conclusion

This study suggested that the predictive models based on the logistic regression and XGBoost algorithm model can predict the occurrence of postoperative SH. The body weight, preoperative PTH, and preoperative ALP are risk factors for SH occurrence after PTX in SHPT patients, while age and preoperative Ca are protective factors for SH. To avoid the occurrence of SH, high attention should be paid to the prevention and treatment of high-risk groups, and preoperative monitoring and management of these indicators should be paid to treat SHPT and related complications better.

## Figures and Tables

**Figure 1:** Flow chart of logistic regression model training.

**Figure 2:** Flow chart of XGBoost algorithm prediction model training.

**Figure 3:** Comparison of clinical data between the SH group and non-SH group in the training set. The difference in clinical data between the two groups was statistically significant (*P* < 0.05).

**Figure 4:** Important feature score in the XGBoost algorithm model.

**Figure 5:** The ROC of the logistic regression model and XGBoost algorithm model in the training set and test set.

**Table 1:** Comparison of general patient data between the training set and test set.

Variable	Training test	Test set	*x* ^2^/*t*	*P*
Age (years)	49.6 ± 7.8	48.7 ± 6.9	-0.519	0.605
Gender (male)	25	11	0.013	0.908
Body mass (kg)	54.7 ± 10.1	53.8 ± 9.3	-0.396	0.693
Dialysis time (years)	5.6 ± 0.5	5.7 ± 0.4	0.920	0.360
Parathyroid gland volume (cm^3^)	4.5 ± 2.1	4.4 ± 2.0	-0.210	0.834

**Table 2:** Comparison of clinical data between the SH group and non-SH group.

Variable	SH group	Non-SH group	*x* ^2^/*t*	*P*
Gender (male/female)	11/7	14/10	0.033	0.856
Dialysis time (years)	7.69 ± 3.43	8.53 ± 3.85	0.897	0.373
Parathyroid gland volume (cm^3^)	4.64 ± 2.16	4.62 ± 2.14	-0.037	0.971
Preoperative P (mmol/L)	2.45 ± 0.51	2.36 ± 0.42	-0.768	0.446

**Table 3:** Multivariate logistic regression analysis of severe postoperative hypocalcemia.

Variable	*β*	SE	*P*	OR	95% CI
Body mass	0.186	4.291	0.032	1.203	1.203~1.428
Age	-0.236	0.070	0.035	1.214	1.219~1.297
Preoperative PTH	0.004	4.215	0.043	1.026	1.006~1.009
Preoperative Ca	-6.608	3.007	0.025	1.062	1.073~1.081
Preoperative ALP	0.027	3.986	0.040	1.031	1.031~1.059

## Data Availability

The data used to support the findings of this study are available from the corresponding author upon request.
